This article has been retracted.

# erbB expression changes in ethanol and 7, 12- dimethylbenz (a) anthracene-induced oral carcinogenesis

**DOI:** 10.4317/medoral.18068

**Published:** 2012-12-10

**Authors:** Luis F. Jacinto-Alemán, Alejandro García-Carrancá, Elba R. Leyba-Huerta, Edgar Zenteno-Galindo, María D. Jiménez-Farfán, Juan C. Hernández-Guerrero

**Affiliations:** 1 Immunology Laboratory, Postgraduate and Research Division, Dental School, National Autonomous University of Mexico, Mexico, D.F., Mexico; 2 Biomedic Cancer research, Biomedic Reseach Institute, National Autonomous University of Mexico & National Cancer Institute, Health Ministry. México, D.F., Mexico; 3 Oral Pathology Laboratory, Postgraduate and Research Division, Dental School, National Autonomous University of México, México, D.F., Mexico; 4 Biochemestry department, Medicine School, National Autonomous University of México, México, D.F., Mexico

## Abstract

Objetive: The aim of this study was to determine erbB expression in normal mucosa, oral dysplasia, and invasive carcinomas developed in the hamster’s buccal pouch chemical carcinogenesis model. Study design: Fifty Syrian golden hamsters were equally divided in five groups (A-E); two controls and three experimental group exposed to alcohol, DMBA, or both for 14 weeks. Number of tumors per cheek, volume, histological condition, erbB expression were determined and results were analyzed by the Mann–Whitney U and Dunn’s test. Results: Control groups and those exposed to alcohol (A, B and C respectively) only presented clinical and histological normal mucosa; while those exposed to DMBA or DMBA plus alcohol (D and E groups) developed dysplasia and invasive carcinomas. erbB2, erbB3, and erbB4 increased their expression in alcohol-exposed mucosa, dysplasia, and invasive carcinomas. We observed a similar expression level for erbB2 in dysplasia and carcinomas; while, erbB3 and erbB4 were similar only in carcinomas. Conclusion: The DMBA and alcohol can be considered as carcinogen and promoter for oral carcinogenesis. The erbB expression is different according to their histological condition, suggesting differential participation of the erbB family in oral carcinogenesis induced by alcohol and DMBA.

** Key words:**erbB, 7,12- dimethylbenz(a)anthracene, oral squamous cell carcinoma.

## Introduction

Worldwide, approximately 274,300 new cases and 127,500 deaths have been attributed to oral cancer during 2002 (1). Oral squamous cell carcinoma (OSCC) is the most frequent neoplasm in the mouth, and many OSCC are preceded by leukoplakia and erythroplakia, which could present epithelial dysplasia (ED), an indicative of malignancy development (2). 7,12-dimethylbenz(a)anthracene (DMBA), a polycyclic aromatic hydrocarbon has been found in high concentration (40-100 ng per cigarette) in the tar fraction of cigarette smoke (3). In mammalian cells, DMBA is bioactivated to the diolepoxide metabolite, which subsequently promotes adducts to adenine and guanine residues in DNA (4). Another important compound is the ethanol, however, the ethanol carcinogenic effect is controversial; some reports consider it as co-carcinogen and/or tumor promoter (5,6). Nevertheless, ethanol consumption has been associated to a 2- to 3-fold increased risk for cancer in the oral cavity, pharynx, larynx, and esophagus (7).

The cellular and molecular analysis, had improve our understanding of OSCC. The analysis of the tyrosine kinase erbB family receptors (erbB1/EGFR, erbB2/Neu/HER2, erbB3/HER3, and erbB4/HER4) had indicated their participation in embryogenesis, proliferation, differentiation, and malignant transformation of breast, renal, colon, and oral cancer. These receptors are activated upon ligand-induced receptor dimerization and, consequently, numerous dimmers are formed, promoting downstream transduction pathway activation, such as MAPK, PI3K, and STAT (8). erbB1 and erbB2 over-expression plays a significant role in driving cancer cells through the cell cycle checkpoints in G1-S transition. erbB2, erbB3, and erbB4 signaling has been associated with apoptosis evasion, invasion, metastases to lymph nodes and angiogenesis (9,10). Specific determination of erbB expression to each tumor could improve our understanding of their biological behavior. Our hypothesis is that erbB receptor expression changes is according to histological condition, for that reason, the aim of this study was to determine the relationship of erbB expression in normal mucosa, dysplasia, and invasive carcinomas developed in the hamster buccal pouch chemical carcinogenesis model.

## Material and Methods

-Population, clinical and histological analysis

Fifty male Syrian golden hamsters (Mesocricetus auratus), 5-week-old, were employed following the guidelines of the Ethics committee of the Postgraduate and Research Division, Dental School, National Autonomous University of México. All animals were housed at four animals per cage, with 12 h light:dark cycles. At 8-week-old animals were divided randomly in five groups; ten animals for each group (A to E groups). The weight of each animal was measured weekly. Animals from group A remained untreated while those in group B received mineral oil (Sigma-Aldrich, M8410, St. Louis, MO) on the right cheek pouch applied three times per week during fourteen weeks at 10 a.m., using a camel’s hair brush No. 4. The animals from groups C and E were left to consume ethanol solution at 15% (Mallinckrodt Baker, V568, Xalostoc, Mexico) ad libitum, consumption was measured two times per week. Groups D and E received DMBA (Sigma-Aldrich, D3254) at 0.5%, dissolved in mineral oil, as above. The amount of carcinogens delivered to each animal was quite uniform using the ‘‘wiped-brush’’ method (11). All animals were simultaneously sedated and killed by a chloroform overdose (Sigma-Aldrich, C2432). The right cheek pouch was dissected and washed in Hank’s balanced salt solution (Gibco-BRL, Cat. 0-125 Pailey, Scotland, UK). Tumor per cheek pouch and two diameters from each tumor were registered. Tumor volume was calculated through diameter measures and the equation V = a x b2 x 0.52; where a is the largest diameter and b is the largest diameter perpendicular to a (12). The cheek pouch was divided in two halves; a portion was fixed in 4% paraformaldehyde solution for 24 h for its histological and immunohistochemical analysis. Another portion was immediately frozen in liquid nitrogen and stored at -80ºC until their western blot analysis.

The fixed samples were processed for paraffin embedding, 4 µm serial sections, and hematoxylin and eosin staining for histopathological analysis was made. The histological classification in normal mucosa, epithelial dysplasia (ED; mild, moderate and severe), and OSCC (well differentiated, WD; moderately differentiated, MD and poorly differentiated, PD) was performed by an oral pathologist.

-Western blot (WB) analysis

Frozen samples were homogenized and lysed in 300 µl of lysis buffer (225 mM saccharose, 10 mM Tris, 0.3 mM ethylene glycol tetraacetic acid, 1% Triton X-100, 2 mM sodium orthovanadate, 10 mM sodium fluoride, 1 mM sodium carbonate; and a mixture of proteinase inhibitors, including 1 mM phenymethylsulfonyl fluoride, 10 µg/ml aprotinin, 5 µg/ml leupeptin, 5 mM benzamidine, 10 µg/ml phenantrholine; BD, Bioscience Pharmigen). Tissue lysate was cleared by centrifugation at 10,000 rpm at 4ºC for 10 minutes. Protein content was quantified using Lowry’s protein assay (13). Protein (25 µg) was electrophoresed in a 10% gradient SDS-PAGE for 120 minutes at 150 mV. The resolved protein was transferred to nitrocellulose membranes (Bio-Rad, Hercules, CA). The membrane was blocked with PBS-1% Triton with 5% non-fat dry milk for 2 h for posterior overnight primary antibodies incubation (erbB1, sc-03, rabbit polyclonal, 1:1000; erbB2, sc-7301, mouse monoclonal, 1:1000; erbB3, sc-285, rabbit polyclonal, 1:1500, and erbB4, sc-283, rabbit polyclonal, 1:1000, all antibodies from Santa Cruz Biotechnology, Santa Cruz, CA) in heat sealed plastic bags at 4ºC. Horseradish peroxidase-labeled (goat anti-mouse sc-2005, mouse anti-rabbit, sc-2357, mouse anti-goat, sc-2354, Santa Cruz Biotechnology) secondary antibodies were used for 1 h at room temperature incubation. The immune complex was visualized using the ECL Western blot detection system (Amersham Pharmacia Biotech, Arlington Heights, IL) according to manufacturer’s instruction. Membranes were exposed one minute to Kodak Biomax light film (Eastman Kodak, Co., Rochester, NY). ß-actin and GAPDH (Sigma A1978, mouse monoclonal, IgG1, 1:2000 and sc-20357 goat polyclonal, 1:1500, Santa Cruz Biotechnology, respectively) detection was used as charge control. The film was scanned for densitometric analysis using Scion Image software (Scion, Frederick, MD). Each representative sample according to histological condition was analyzed in triplicate.

-Immunohistochemistry (IHC)

The IHC analysis for erbB1, erbB2, erbB3, and erbB4 was performed according to reported (14). Eight slides for each sample were deparaffinized and rehydrated in xylene and alcohol washes. Antigenic retrieval in 10 mM citrate buffer; endogenous peroxidase blockade in 3% hydrogen peroxide, unspecific blockade with serum-free protein block (DakoCytomation, Dako, Carpinteria, CA) and posterior immersion in 0.2% Triton X100 were performed. Four slides were incubated overnight with anti-erbB primary antibodies at 4°C in 1:100 dilution. Biotinylated link universal secondary antibody and streptavidin-HRP incubation for 30 minute each were performed (Dako, Carpinteria, CA). Posterior 3,3’diaminobenzidine revealing (Dakocytomation, Dako, Carpinteria, CA) and Hill’s hematoxylin nuclear counterstaining were done, for posterior dehydration in alcohol-xylene serial washes and mounting with hydrophobic resin (14). For negative control (the rest four slides), the primary antibody was substituted by phosphate buffer saline (PBS) solution. From each slide, a digital photomicrograph of 2000 × 1500 pixels was obtained at 1000X magnification with a digital camera (Olympus C-3040 Tokyo, Japan). Cellular expression zone was determined semiquantitatively as follows: zone (membrane, cytoplasm, and nucleus) and percentage of positive cells (0 = 0% cells, 1 = 1 to 29% cells, 2 = 30 to 69% cells, and 3 = >70 % cells).

-Statistical analysis

All data are presented as means ± SE. Mean values were analyzed by ANOVA with a post hoc Mann–Whitney U and Dunn’s test to compare differences between groups and similar histological conditions. Statistical significance was at P < 0.05, SPSS v.13.0. Software package (SPSS Inc., Chicago IL) was used for statistical analysis.

## Results

-Clinical and histological analysis

The final population was 47 hamsters; in groups D and E two and one animal were lost by territorial disputes, respectively. The mean weight of all specimens was of 99.2 ± 6.6 g, none important variation was observed. The alcohol consumption for C and E groups was 20.4 ± 2ml and 18.9 ± 2.3ml, respectively. In clinical examination, only D and E groups developed tumors. The number of tumors per cheek in D group was of 3.2 ± 1.7 with a mean volume of 15.4 ± 9.8 mm3; animals of group E showed 2 ± 0.7 tumors with a mean volume of 84.6 ± 44.9 mm3.

The histological analyses indicate that all specimens of A, B, and C groups showed normal mucosa. Group D showed four speci-mens diagnosed as severe ED and 4 WD OSCC. The E group presented two specimens classified as severe ED, 5 WD OSCC, one MD OSCC and one PD OSCC.

-erbB expression

The WB analysis indicates that erbB1 did not present changes in expression in normal mucosa of groups A, B, and C. The severe ED and WD OSCC developed in D and E groups revealed noticeable variation between similar histological condition and comparing to control normal mucosa. erbB2 showed a significant increase (P = 0.04) in alcohol-exposed mucosa compare to control normal mucosa. In severe ED showed similar expression patterns, while WD OSCC of E group showed significant increase. erbB3 presented significant changes in alcohol-exposed mucosa (P = 0.01), severe ED and WD OSCC compare to control; since, only severe ED showed significant difference between similar histological condition. erbB4 showed variation in severe ED and WD OSCC compare to control; since, comparing similar histological condition only severe ED showed significant variation in their expression ( Table 1), (Fig. 1).

**Table 1:** erbB expression analysis according their histological condition.

**Figure 1:** Expression of erbB family members in oral carcinogenesis. a) Western Blot analysis according to histological condition. erbB1 showed similar expression for normal mucosa (1 to 3) and different expression for severe ED and carcinomas. erbB2 increase their expression in alcohol exposed mucosa, severe ED and carcinomas. 1) Normal mucosa group A, 2) Normal mucosa group B, 3) Normal mucosa group C, 4) Severe ED group D, 5) Severe ED group E, 6) WD OSCC group D, 7) WD OSCC group E, 8) MD OSCC group E and 9) PD OSCC group E. b) IHC analysis. a) erbB1 expression in normal mucosa with predominant membrane expression pattern b) erbB1 in WD OSCC of group D with cytoplasm expression pattern, c) erbB2 expression in normal mucosa of group A showed cytoplasm expression pattern without presence in corneous stratum, d) erbB2 expression in WD OSCC of group D with cytoplasm expression pattern even in cells next to keratinization area, e) erbB3 expression in normal mucosa, f) erbB3 expression in alcohol exposed mucosa, it shows an important expression increase, g) and h) showed similar expression pattern of erbB4 in WD carcinomas of D and E groups. Objective 100X. Scale bar = 8 µm

-Cellular expression zone 

To determine the cellular expression zone IHC analysis was performed. We observed that erbB1 in normal mucosa (A to C groups) was expressed predominantly in membrane, however, severe ED and all OSCC showed differential expression patterns compare to normal mucosa and between similar histological conditions. erbB2 presented cytoplasm expression in all normal mucosa and increase their membrane expression in severe ED and WD carcinoma, with a similar expression pattern between similar histological condition. erbB3 and erbB4 presented variation in alcohol-exposed mucosa, severe ED and WD carcinomas compared to control normal mucosa, and differential expression between similar histological condition ( Table 2), (Fig. 1).

**Table 2:** erbB expression according to their cellular zone.

## Discussion

Alcohol and tobacco consumption are very common in some areas of the world, this behavior increases the relative risk to develop larynx, pharynx, esophagus, and oral cancer (3-6,15). We confirm above, when observed that alcohol, DMBA and both exposure induced clinical, histological, and molecular alterations related to oral carcinogenesis. DMBA is an organ-specific carcinogen, which can mediate neoplasm transformation by inducing DNA damage, generating excess reactive oxygen species, mediate the chronic inflammatory process and tumor develop (16). Our results from D and E groups are according with that above, however, the tumors developed in animals receiving DMBA and alcohol (group E) were bigger than those from animals receiving only DMBA (D group); this would be associated to alcohol’s promoter effect (17). Nevertheless, the promoter effect of alcohol is controversial, some reports attribute this to its metabolic product, acetaldehyde, because that interferes with DNA synthesis and repair, induces point mutation, sister chromatin exchanges, and chromosomal aberration (5,18). Another possible promoter effect derived from alcohol is the increase in mucosa’s permeability to toxic and carcinogenic compounds, it has been reported that diluted ethanol (15%) may be more effective than higher concentration of ethanol, because, this concentration allows molecules and compounds to cross the membrane (19). Both possible effects could induced malignant transformation, however to confirm the malignant phenotype a histological analysis is required. The histological analysis of A, B and C groups showed normal mucosa, D group developed severe ED and WD carcinoma, whereas group E also presented ED, however, invasive carcinoma was the predominant histological condition. This could be compared to patients that consume both compounds, in whom the relative risk to develop oral carcinomas is higher with ethanol and tobacco consumption (15). The golden Syria Hamster chemical oral carcinogenesis is a model that closely resembles a human oral tumor, both histologically and morphologically. Lipid peroxidation, epigenetic control, angiogenesis and apoptosis had been analyzed; however, the implication of an important receptor family, as erbB, during sequential pathogenesis of this model had not been reported (16,20-22).

The role of erbB receptors in carcinogenesis has been established in breast, colon, lung cancer, and head and neck carcinoma. Their expression and function analysis is an important research issue because the possible approaches could be applied in specific therapies (10). Our results indicate that erbB1 showed similar level and pattern expression in normal mucosa; and variations in its level and zone expression in severe dysplasia and invasive carcinomas developed in D and E groups. The above suggest that erbB1 expression is necessary in histological normal condition, but when an early or severe malignant transformation is present the level and cellular zone expression can modify. An interesting feature was the change in expression zone of membrane to cytoplasm in dysplasia and carcinomas as compared to normal mucosa. Lin et al. have reported that erbB can translocate from membrane to nucleus promoting transcription, and enhancing malignant transformation (23). It is possible that this effect is carrying out, nevertheless, to determinate what are the particular mechanism involved, transcription or proteomic analysis is necessary.

Some reports suggest that only erbB1 and erbB2 are sufficient to induce cell transformation, however, others indicate that erbB3 and erbB4 could participate (24-26). Our results suggest an increase in erbB2, erbB3, and erbB4 expression in alcohol exposed mucosa, severe ED and invasive OSCC compared to control normal mucosa. It has been reported that perturbation in epithelial permeability barrier leads to increasing mRNA levels of IL-1a, IL-1b, TNFa, and GM-CSF, as well as in the inflammatory re-sponse. The increase of erbB receptors could be a response mechanism that promotes epithelial maintenance, repair, differentiation, and enhancement of survival in exposed cells, however, if a carcinogen appears the malignant transformation could be more possible (19,27).

In our experimental model erbB2 showed level expression increase in alcohol exposed mucosa, severe ED and carcinomas, with similar membrane cellular expression only for severe ED and well differentiated OSCC. This result agrees with the report by Fong et al., which indicated that erbB2 expression in normal mucosa was almost undetectable, very low in ED, and significantly higher in OSCC, suggesting the participation of this receptor in early transformation (26). Respect to erbB3 a similar level expression pattern to erbB2 was observed in alcohol exposed mucosa, severe ED and carcinomas; however, in their cellular zone expression a heterogeneous pattern was observed. Xia et al. have reported that principally erbB2 and erbB3 expression to be associated to malignant phenotype, suggesting that these receptors may help predict the outcome of patients with OSCC (25). However, our results in this animal model suggest that erbB4 and erbB2 are the predominant receptors in well differentiated OSCC. These changes could be derivate from reduction of erbB1 expression, heterogeneous erbB3 expression and molecular structure of erbB4. The role of erbB4 in neoplasm biology is controversial, because some reports suggest a protector action for this receptor and other consider it as an indicator of aggressiveness and metastasis (24,25,28-30). Today, the golden Syrian hamster model is an important tool in the oral cancer research; nevertheless, the compare to human cancer is necessary, in our opinion this is the principal limitation of that experimental model. Until one does not demonstrate similarities between both carcinogenic processes, the applications will be reduced.

The understanding of cellular and molecular carcinogenesis, could give to us the possibility of restrain the advance of malignant transformation using specific inhibitors, monoclonal antibodies or chemopreventive compounds directed to erbB2, erbB3 or erbB4. The above means a promising advance in oral oncology because currently many young people consume ethanol, tobacco or both and the oral cancer risk is increasing. In this study we observe the carcinogenic potential of DMBA, the promoter effect of ethanol and the particular behavior of erbB receptors, suggesting a homogenous pattern for erbB2 and erbB4 in well differentiated carcinomas. The underlying revelation of the mechanism involved is necessary to lead to the application of new therapeutic strategies derived from this knowledge.
